The article "The Occurrence and Distribution of Plasmodium Species in Woyn Wuha Health Center, Ethiopia" was published in 2022. Journal: Biomed Res Int.

# The Occurrence and Distribution of Plasmodium Species in Woyn Wuha Health Center, Ethiopia

**DOI:** 10.1155/2022/2881879

**Published:** 2022-09-05

**Authors:** Anmut Assemie

**Affiliations:** Department of Biology, Wachemo University, PO Box 667, Hossana, Ethiopia

## Abstract

*Plasmodium* species is an important causative agent of malaria in the world including Ethiopia, and the majority of people were at risk of infection. The study's general objective was to determine the occurrence and distribution of *Plasmodium* species in the study area through microscopic examination of blood films. A cross-sectional study was carried out in the study sites from September 2016 to February 2017. Out of 512 participants, 32 (6.25%) were malaria positive. Of these, 17 (53.12%, 95% CI: 0.358, 0.704) were *P. vivax*, 12 (37.5%, 95% CI: 0.207, 0.543) *P. falciparum*, and 3 (9.375%, 95% CI: -0.007, 0.195) mixed out of the total positive case. The occurrence of parasites was greater in rural villages (59.375%) than in urban villages (40.625%) but not significant (*χ*^2^ = 1.2917, *df* = 1, *p* = 0.2557). More males were infected compared to females but not significant (*χ*^2^ = 0.0005665, *df* = 1, *p* = 0.981). The monthly distribution of *Plasmodium* species was higher in September and October but there was no significant variation in each month (*χ*^2^ = 10.142, *p* = 0.4281). Due to the high occurrence of *Plasmodium* vivax in the study area, the result contrasts with the national figure of the *Plasmodium* species report. The result of the current study may be useful to those individuals who work in *Plasmodium* species control and prevention program.

## 1. Introduction

Malaria is caused by protozoan parasites of the genus *Plasmodium*, which is one of the world's major causes of illness and death. Malaria is a disease that affects over 97 nations and affects about 44% of the world's population. Malaria causes 216 million illnesses and 445,000 deaths worldwide, with the African region accounting for over 90% of cases and fatalities. In addition, 14 sub-Saharan African nations and India accounted for 80% of the worldwide malaria burden [1].

*Plasmodium falciparum* is the most common cause of malaria in Africa [2], but *Plasmodium vivax* is found in a few African nations, including Ethiopia [3] and Uganda [4]. Compared to these two main species, *P. malariae* and *P. ovale* are considerably rarer and largely understudied. *P. ovale* has been found mostly in sub-Saharan Africa [5]. *P. malaria* is widespread in tropical Africa, where coinfections with *P. falciparum* are common [6]. Malaria is a mosquito-borne disease caused by five *Plasmodium* species [1] and transmitted by infective female *Anopheles* mosquito bites [1–3]. *P. falciparum* and *P. vivax* are the most widely distributed and well-known malaria-causing species in Ethiopia, accounting for 60% and 40% of cases, respectively [4]. The distribution of *Plasmodium* species varies according to localities and seasons [5].

In 2015, there were an estimated 212 million cases of malaria and 429,000 deaths worldwide [6]. More than 80% of the cases and 90% of all deaths occur in sub-Saharan Africa, with 77% occurring in children under the age of five [6]. Malaria is the leading cause of morbidity and mortality in Ethiopia; approximately 75% of the landmass is endemic to malaria and about 68% of the total population lives in areas at risk of malaria [7].

This study was designed to generate useful information that is mandatory for malaria control and improve policies and design interventions for malaria prevention. The result will also be useful to evaluate the progress of the district towards achieving the regional and national target to take immediate actions in planning and implementing prevention and control strategies.

## 2. Materials and Methods

### 2.1. Description of Study Area

The study was conducted in °00′19^″^ N and 37°45′ 23^″^ E Woyn Wuha Health Center, Bibugn District, East Gojjam, Ethiopia. The health center is located 108 km and 507 km from Deber Markose town and Addis Ababa, respectively. Woyn Wuha Health Center is located in the South Moseba village, on the west by the West Gojjam Zone Dega Damot district, on the north-west by Dega Damot, and on the east and north by Hulet Eju Enese.

The largest ethnic group reported in the study area was the Amhara. The majority of the inhabitants practiced Ethiopian Orthodox Christianity, with 99.56% reporting it as their religion. Most residents have an agriculture-based economy, particularly teff, maize, and wheat being the main products.

### 2.2. Study Design and Sampling Methods

A cross-sectional study was conducted among patients referring to selected health centers. Patients, who have been referred to health centers during the data collection period, were randomly selected from the study area, for any kind of health service, as the study population. The samples were obtained from September 2016 to February 2017 at the selected health center.

### 2.3. Sample Size Determination

Since there were no previous studies concerning the abundance and distribution of Plasmodium species in the area, 50 : 50 was assumed for prevalence (*P*). So the required sample size was calculated using a formula for a single population proportion at a 95% CI level (*Z*ά/2 = 1.96). A minimum of 384 samples (*n*) was generated using a 5% marginal error (*d*) as shown in the following:

(1) $$\begin{array}{c} n=Z^{2}P\frac{1-P}{d^{2}},\\ n=\left(\frac{\left(Z^{2}\left(ά/2\right)\right)\left(50\%\right)\left(50\%\right)}{d^{2}}\right),\\ n=\frac{\left(1.96\right)\cdot \left(1.96\right)\cdot \left(0.5\right)\cdot \left(0.5\right)}{{\left(0.05\right)}^{2}},\\ n=384, \end{array}$$

where *n* is the sample size, *P* is the average prevalence, *Z*ά/2 is the *p* value at 95% CI from the table, and *d* is the worst accepted value/marginal error.

Therefore, once the minimum number of samples was obtained, by adding a 25% contingency nonresponse rate, a total of 512 study subjects were enrolled.

### 2.4. Blood Sample Collection and Parasite Identification

The parasitological examination was performed by experienced technicians of the health center among the people who visited the health center for all services.

A small blood volume was collected from the cases. Two blood slides each composed of thick and thin films were prepared for each participant by a medical laboratory technician according to the standard operating procedure [8]. Slides were labeled and air-dried horizontally in a slide tray, and thin films were fixed with methanol after drying. Slides were stained with 3% Giemsa for 30-45 minutes at each health center laboratory unit [9]. Blood slides were read and cross-checked by senior laboratory technologists at the laboratory unit, as either negative for blood parasites, *P. falciparum* positive, *P. vivax* positive, or mixed infection with both. The staining technique and blood film examination were conducted according to the standard of WHO protocols [10, 11].

### 2.5. Ethical Clearance and Study Participants

Ethical approval of the study was obtained from Debre Markos University College of Natural Science, and the collection of blood sample from participants was allowed by Woyn Wuha Health Center's office director. Positive patients were treated with coartem for *P. falciparum* and chloroquine for *P. vivax.* They have given written and verbal consent to take part in the study after an adequate explanation of the significance of the study. Besides, the potential harm and benefit of the study were explained to the respondents. Only volunteer sample populations with informed consent were included in the study. Participants who were under 18 years of age were included in the study after obtaining written consent from the parent/guardian.

### 2.6. Data Analysis

All the data that are collected during the study period are summarized by a table and expressed by percent. Data collected on blood film examination and associated parasites were entered and analyzed using SPSS version 20.0 statistical software. Plasmodium species distribution between urban and rural villages and sociodemographic was compared using the chi-squared test. Results were considered to be statistically significant when *p* value was <0.05.

## 3. Results

### 3.1. Sociodemographic Characteristics of the Participants

A total of 512 respondents were included in the study, of which 357 were from rural villages and 155 were from urban villages. Of these, 329 were males and 183 were females as shown in Table 1. The vast majority of study participants were male and rural in residence.

### 3.2. The Prevalence of Malaria

Out of the total study participants, 32 were malaria positive. Of the total positive case, 62.5% males and 37.5% females were malaria positives. The greatest prevalence was in the 15 and above age group, 22, compared to less than 5 years and in the age group between 5 and 14. There was no statistically significant variation between malaria infection and age, residence, and sex of the participants (*χ*^2^ = 0.39096, *df* = 2, *p* = 0.8224), (*χ*^2^ = 1.2917, *df* = 1, *p* = 0.2557), and (*χ*^2^ = 0.0005665, *df* = 1, *p* = 0.981), respectively, as indicated in Table 2. The abundance of *Plasmodium* species in rural villages was much greater than in urban areas.

### 3.3. Occurrence and Distribution of Plasmodium Species

The total number of parasite-positive slides from the studied locations was 32 cases, of which 19 cases (59.375%) were related to a rural area, and 13 cases (40.625%) were related to an urban area. Of the total number of positive parasites, 3.71% were in rural villages and 2.54% were in urban villages as shown in Table 3.

In the current research, *P. vivax* 17 (53.125%), *P. falciparum* 12 (37.5%), and mixed 3 (9.375%) are the three *Plasmodium* species identified. The result showed that *P. vivax* species was the most prevalent *Plasmodium* species in the study area. From the total number of positive *Plasmodium*, the majority of them were males, and the females were in minority. From these, 13 males were positive for *P. vivax* and 5 were positive for *P. falciparum*, whereas 4 females were positive for *P. vivax* and 7 were positive for *P. falciparum.* The distribution of *Plasmodium* species with sex was not significant (*χ*^2^ = 3.661, *df* = 1, *p* = 0.1604). The highest prevalence of malaria was seen in the age group of ≥15 years, which is 22 of 329 individuals. The least positivity was seen in the age group of <5 years which is 3 of the total 47 examined individuals. In the majority of the age group, the dominant *Plasmodium* species is *P. vivax* as present in Table 4.

Among the total diagnosed with *Plasmodium* species from September 2019 to February 2020, 32 (6.25%) were slide-positive. Monthly distribution of *Plasmodium* species was not significant (*χ*^2^ = 10.142, *df* = 10, *p* = 0.4281). But the number of suspected and confirmed cases showed a fluctuating pattern in the months studied as indicated in Figure 1. Based on the current studies, the highest numbers of cases, 11 (34.375%) and 9 (28.13%), were registered in October and September, respectively, during the rainy season. The remaining 12 (37.5%) of the cases were observed during the semidry and dry months from November to February. The lowest number of confirmed cases was recorded in January and February.

## 4. Discussion

The current study was conducted to evaluate the occurrence and distribution of *Plasmodium* species and to map out areas of high *Plasmodium* in the study area. The prevalence of *plasmodium* species in the present study was 6.25%. So the occurrence of the *Plasmodium* species in the current studies was lower than in the study conducted in Ataye, North Shoa (8.4%) [12], South Wollo (7.52%) [13], Metema Hospital (17%) [14], Koladiba Health Center (39.6%) [15], Woreta Town, Amhara Region (32.6%) [16], Adi Arkay Health Center, North Gondar Zone (36.1%) [17], Tselemti Wereda, North Ethiopia (28.1%) [18], East Shewa Zone of Oromia Regional State, Ethiopia (25%) [19], Kalala Health Center in Haro Limmu Woreda, East Wollega Zone, Western Ethiopia (49.4%) [20], Dilla town and the surrounding rural areas, Gedeo Zone, Southern Ethiopia (16%) [21], and Goljota health center, Heben Arsi District, West Arsi Zone, Oromia Regional State, Ethiopia (14.8% in 2012, 21.4% in 2013, 14.2% in 2014, 12.9% in 2015, and 13.2% in 2016) [22]. And this is also lower than the systematic review and meta-analysis conducted on malaria prevalence among adults, children, and pregnant women in Ethiopia, which results in 13.61%, 9.07%, and 12.72%, respectively [23–25] but higher than the studies conducted in the Butajira area, south-central Ethiopia (0.93%) [26], Oromia and Southern Nations, Nationalities, and Peoples' Region (SNNPR) regions (2.4%), and Amhara Regional state (4.6%) [27, 28], and partially similar to the studies conducted in Benna Tsemay district of pastoralist community, Southern Ethiopia (6.1%) [29] and Dembia district, Northwest Ethiopia (6.7%) [30].

This difference might be due to the variation in the intensity of vector control strategies, altitude, microclimate, community awareness about malaria prevention and control methods, habitat modifications and the ability of the laboratory professionals to detect *Plasmodium* species correctly, methods of diagnosis, nature of participants, and sample size.

The identified *Plasmodium* species in the present study were *P. vivax*, *P. falciparum*, and mixed 3.32%, 2.34%, and 0.59%, respectively, out of the total parasite-positive participants. In this case, *P. vivax* was the most abundant *Plasmodium* species consisting of 53.125% of the total positive cases in the study area during the study period. This study was related to the study conducted in Hallaba Health Center, Southern Ethiopia, where 119 people (70.41%) were infected with *P. vivax*, 39 people (23.08%) with *P. falciparum*, and 11 people (6.51%) with mixed infection [31], Chichu and Wonago Health Centers, South Ethiopia (*P. vivax* (52.75%, *P. falciparum* (35.16%), and mixed (12.09%)) [32]. The overall estimated distribution of *P. falciparum* and *P. vivax* in the current study was similar with [33–41] and contradict with other [21, 26, 31, 32, 42–46].

The prevalence of *P. vivax* was also higher in males than in females. The reason behind this result should be that males commute to different malaria-risk areas of Ethiopia for daily labor and they might caught (positive) it there and relapse when they came to this study area due to the relapsing behavior of *P. vivax*.

These studies contrast the study conducted in the Jimma zone at Assendabo health center [47], which shows the prevalence of *P. vivax* at 45.7% and *P. falciparum* at 54.3%, Kalala Health Center in Haro Limmu Woreda, East Wollega Zone, Western Ethiopia (54.5%, 15.8%, and 6.6% were infected with *P. falciparum*, *P. vivax*, and mixed, respectively) [20].

The finding in the study area, where the highest prevalence was in the age group 15 years and above, does not fit into the conventional characterization of *Plasmodium* species distribution based on age stratification, contrary to the established convention that infection among children less than 5 years old in stable communities implies autochthonous malaria transmission [37].

The local variation in malaria prevalence in Ethiopia is exacerbated further by the local variance revealed in this study, which found that the prevalence was much greater in rural Kebeles than in urban areas. In the current research, the highest malaria case was recorded in September and October, which is consistent with the findings [38]. Therefore, the relatively high transmission that occurs in September and October, following the heavy rains, was to be expected in the study area.

In the present study, the distribution of *Plasmodium* species in males was higher than in females in all study seasons in the study area. The reason behind the variation of *Plasmodium* species abundance was maybe, in the study area, males spend the majority of the night working outside the house where they might be easily baited by malaria vectors which are active at night, but most females spend most of the time inside the house. So they were not at risk of malaria in the study village.

## 5. Conclusion

The current study was the first in the study area, concerning the occurrence and distribution of *Plasmodium* species in the selected villages. Based on the finding of the study, the three *Plasmodium* species that cause malaria were *P. falciparum*, *P. vivax*, and mixed. Out of the three *Plasmodium* species identified during the study period, *P. vivax* was higher in prevalence and more abundant in September and the rural village than *P. falciparum* and mixed. The highest occurrence and distribution of *Plasmodium* species was recorded in the age group ≥15. Generally, the abundance and distribution of *P. vivax* and *P. falciparum* are different from the national figure.

## Figures and Tables

**Figure 1:** Monthly distribution of *Plasmodium* species.

**Table 1:** Sociodemographic characteristics of the study participants.

Variables		Study participants	%
Sex	Male	329	64.26
	Female	183	35.74

Residence	Rural	357	69.73
	Urban	155	30.27

Age	<5	47	9.18
	5-14	136	26.56
	≥15	329	64.26

Total		512	100

**Table 2:** Malaria prevalence based on the sociodemographic.

Variables		Number examined	Malaria positive			
			Positive	Negative	*χ* ^2^	*p* value
Sex	Male	329	20	309	0.0005665	0.981
	Female	183	12	171		

Residence	Rural	357	19	338	1.2917	0.2557
	Urban	155	13	141		

Age	<5	47	3	44	0.39096	0.8224
	5-14	136	7	129		
	≥15	329	22	307		

Total		512	32	480		

**Table 3:** Overall malaria infection prevalence in two villages.

Villages	Sex	No. of examined	No. of positive	%
Rural	Male	187	13	2.54%
	Female	120	6	0.97%

Urban	Male	142	7	1.37%
	Female	63	6	0.97%

Total		512	32	6.25%

**Table 4:** Distribution of *Plasmodium* species.

Variables		Total examine	Presence of *Plasmodium* species					
			*P. falciparum*	*P. vivax*	Mixed	Total	*χ* ^2^	*p* value
Sex	Male	329	5	13	2	20	3.661	0.1604
	Female	183	7	4	1	12		
	Total	512	12	17	3	32		

Residence	Rural	357	4	12	3	19	6.3126	0.04258
	Urban	155	8	5	0	13		
	Total	512	12	17	3	32		

Age	<5	47	2	0	1	3	5.3754	0.25095
	5-14	136	2	5	0	7		
	≥15	329	8	12	2	22		
	Total	512	12	17	3	32		

## Data Availability

All the data used to support the findings of this research are included in the manuscript.
